# Prediction of Pulmonary Fibrosis Based on X-Rays by Deep Neural Network

**DOI:** 10.1155/2022/3845008

**Published:** 2022-03-26

**Authors:** Da Li, Zhuo Liu, Lin Luo, Siyu Tian, Jingyuan Zhao

**Affiliations:** ^1^Dalian University of Technology, Dalian 116024, China; ^2^The First Affiliated Hospital of Dalian Medical University, Dalian 116011, China; ^3^The Second Affiliated Hospital of Dalian Medical University, Dalian 116000, China; ^4^Dalian Medical University, Dalian 116044, China

## Abstract

As a fatal lung disease, pulmonary fibrosis can cause irreversible damage to the lung, affect normal lung function, and eventually lead to death. At present, the pathogenesis of this kind of disease is not completely clear, and there is no radical cure. The main purpose of the treatment of this disease is to slow down the deterioration of pulmonary fibrosis. For this kind of disease, if it can be found early, it can be treated as soon as possible and the life of patients will be prolonged. Clinically, the diagnosis of pulmonary fibrosis depends on the relevant imaging examination, lung biopsy, lung function examination, and so on. Imaging data such as X-rays is a common examination means in clinical medicine and also plays an important role in the prediction of pulmonary fibrosis. Through X-ray, radiologists can clearly see the relevant lung lesions so as to make the relevant diagnosis. Based on the common medical image data, this paper designs related models to complete the prediction of pulmonary fibrosis. The model designed in this paper is mainly divided into two parts: first, this paper uses a neural network to complete the segmentation of lung organs; second, the neural network of image classification is designed to complete the process from lung image to disease prediction. In the design of these two parts, this paper improves on the basis of previous research methods. Through the design of a neural network with higher performance, more optimized results are achieved on the key indicators which can be applied to the real scene of pulmonary fibrosis prediction.

## 1. Introduction

Pulmonary fibrosis is also known as interstitial lung disease which is a chronic progressive interstitial lung disease because a large number of fibroblasts continue to proliferate leading to lung inflammation and then leading to changes in lung tissue structure [1]. Generally speaking, it refers to the formation of scar tissue in the process of repair after the normal lung tissue is damaged. Scar thickens lung interstitium which makes it difficult for oxygen to pass through alveoli and enter the blood. Therefore, the clinical manifestations of patients in the middle and late stages will have difficulty in breathing and hypoxia. Pulmonary fibrosis is a type of disease that is almost impossible to be cured. This type of disease is also called tumor-like disease. Once diagnosed, it is necessary to receive long-term or even lifelong treatment [2]. The main purpose of current clinical treatment is to control and delay the progress of the disease, make the disease no longer worsen, maintain the normal lung function of patients, and prolong the life of patients. Early interventional treatment is of great significance to prolong the life of the patient. Therefore, a rapid and accurate diagnosis is particularly important.

The clinical manifestations of patients with pulmonary fibrosis disease are not significant in the early stages of the disease. However, with the rapid development of the disease, the patients will experience respiratory failure in a short period of time. For this kind of disease, the earlier the diagnosis and treatment, the longer the survival time; clinically, the main diagnostic methods for pulmonary fibrosis include lung imaging, lung tissue biopsy, and lung function check. The accuracy of reliance on lung medical imaging to diagnose such diseases depends on the relevant high-precision radiology imaging equipment and is also limited by the experience and knowledge of the radiologist and the attending doctor. Even doctors in related professions may still have deviations in their judgments on this disease. For the same case, different doctors have different diagnosis opinions and results. The objective judgment of the computer has a huge effect on correcting these subjective errors. If the computer can be used to assist in the diagnosis of related examination results, it will play a role in the diagnosis of such diseases in a timely manner which is of great significance value for both doctors and patients.

## 2. Prediction of Lung Fibrosis Based on X-Rays

### 2.1. Basic Model Design

X-ray film is a two-dimensional picture formed by X-rays penetrating human tissues and organs after penetrating a human body or an object and projecting on a specific negative film which can visually observe the lesions in different positions. Chest X-ray examination is one of the most common and cost-effective medical imaging examinations in clinical practice. In 2017, the NIH Clinical Center released a dataset containing more than 100000 chest X-ray images and corresponding labels for use by researchers all over the world, namely, the chest X-ray 14 dataset [3]. The chest X-ray 14 dataset contains 14 types of chest diseases including pulmonary nodules, fibrosis, and emphysema. Therefore, on this public data set, we use the data of its fibrosis part to predict the classification of lung fibrosis. Wu Enda's team once proposed the CheXNet network framework on the basis of this data set [4–6] which claimed to have reached a level far surpassing professional radiologists. CheXNet is essentially a 121-layer DenseNet network. By adding a full connection layer, after multiple convolution operations, it achieves accurate prediction and classification of multiple lung diseases.

Therefore, the basic model draws on its related ideas and will make related improvements on the basis of the DenseNet network to achieve a more accurate prediction and classification of pulmonary fibrosis. Since chest X-ray is a two-dimensional image data, the images of other organs of the chest will also be included when the film is taken. The images of different organs and skeletons overlap with each other and the features of lesions are obviously covered and the differentiation between tissues is small. Therefore, in order to better improve the accuracy of the model before using CheXNet for predictive classification, we segment the image and separate the relevant image parts of the lungs to reduce the impact of other organ images on the final result. To a certain extent, the quality of the classification of images determines the quality of the classification task. High-quality segmentation pictures can enable the model to learn unbiased knowledge and make a more objective evaluation.

In the field of medical image processing, there are two main frameworks for medical image segmentation. One is based on CNN and the other is based on FCN (Full Convolutional Network). We adopt the U-Net network structure improved from the FCN network. U-Net symmetrizes the process of downsampling and upsampling. In addition, by adding skip-connect-related structures, it fuses multidimensional information such as global and local details of the image. Through the fusion of this information, the comparison showed good results. On the basis of U-Net-related networks, different networks such as U-Net++ and V-Net have carried out deeper structural improvements. Through the splicing of high-dimensional semantics and low-dimensional semantics, they can be used in different tasks and both showed good results.

After image segmentation is used to obtain relevant pictures containing only the lung structure, we use the CheXNet network to make relevant predictions on the image. CheXNet is essentially a 121-layer DenseNet network. The DenseNet network was proposed for the first time to connect all inputs to the output layer. This method is called dense connection. The input of each layer comes from the output of all the previous layers. This reduces the overall number of parameters of the model and at the same time suppresses the overfitting situation so that the network can be deeper, but in the training process, the calculation and storage of the intermediate variables are expensive, and there are greater requirements for computing power and memory. The dense connection method is shown in Figure 1.

Corresponding to the structure shown in the figure, the input and output of the non-first layer and the learning of the related network satisfy the following relationship:

(1) $$\begin{array}{c} X_{l}=H_{l}\left(\left[X_{0},X_{1},X\circ_{2}\ldots X_{l-1}\right]\right). \end{array}$$

Among them, [*X*_0_, *X*_1_, *X*_2_ … *X*_*l*−1_] represents the splicing of the feature map output from the 0th layer to the *l* − 1 layer in the channel dimension, *X*_*l*_ represents the output of the *l* layer, and *H*_*l*_ represents the function transformation of the *l* layer.

Since the input of each layer is the splicing of the previous *N* layers in the channel in order to prevent the subsequent network layer from the dimensional explosion on the channel before each convolution operation, the Bottleneck Layer structure is added. The essence of the Bottleneck Layer structure is a convolution of 1 × 1. The model changes the number of feature maps by using the convolution of size 1 × 1. In the same Dense Block, the size of the feature maps is the same, and between different blocks by introducing the Transition Layer structure and also by convolution of 1 × 1, the number of output feature maps is randomly reduced. There is no difference in structure between Transition Layer and Bottleneck Layer. The main difference lies in the number of feature maps and the location used. Before the Bottleneck Layer is used for each convolution, the number of feature maps output is the growth rate in the same block (growth rate) 4 times the growth rate which is the number of feature maps output by the convolution operation in the same block. The Transition Layer is used between the block and the block, and the number of feature maps output by the previous block is randomly reduced by a certain ratio. In this experiment, we added these two structures on the basis of DenseNet; the actual network used is DenseNet-BC. DenseNet-BC absorbs the advantages of DenseNet, and at the same time, it limits the width of the network so that the network can narrow fewer parameters. The network structure of DenseNet-BC is shown in Figure 2.

Due to the splicing method, the memory consumption is relatively large. Therefore, we use the DenseNet-BC network structure with 3 Dense Blocks; the growth rate is 16. The width and depth of the model directly affect the learning effect of the model, and the reduction of parameters causes the model to be inferior to the CheXNet network in terms of related indicators. Generally speaking, the knowledge reasoning and learning ability of wider and deeper network models will be stronger. In Wu Enda's CheXNet network structure, 4 Dense Blocks are used, and the growth rate is also higher than 24. Therefore, the accuracy of the model will be higher.

### 2.2. Basic Model Evaluation and Problem Analysis

Whether it is the upstream U-Net or the downstream predictive model DenseNet-BC, its essence is in two classification-related tasks. Therefore, we all use the cross-entropy loss function to evaluate the performance of the model. The loss function is as follows:

(2) $$\begin{array}{c} \text{loss}=-\sum y_{i}\log\;s_{i}. \end{array}$$

Among them *y*_*i*_ represents the label of the category, a positive example is 1, a negative example is 0, and *s*_*i*_ represents the probability that the prediction is positive. The upstream and downstream tasks of predictive classification experiments related to pulmonary fibrosis diseases based on X-rays are essentially binary classification tasks. Therefore, we can use the binary cross-entropy loss function as the loss function of the model's prediction effect. In order to prevent overfitting of the model in the loss function part, we added the L2 regularization term. Finally, we use the following loss function:

(3) $$\begin{array}{c} \text{loss}=-\left[y_{i}\log\;s_{i}+\left(1-y_{i}\right)\log\left(1-s_{i}\right)\right]+\alpha {\left\|w\right\|}_{2}^{2}. \end{array}$$

Because the chest X-ray 14 does not contain information related to lung segmentation, we used the data sets from [7, 8]. The data set contains more than 700 X-ray images and their corresponding mask images which can be used to describe whether the pixels at the corresponding positions are part of the lung that is the ground truth of each pixel.

We take 20% of the data set as the test set 15% as the verification set and the rest as the test set. The dataset contains the classification of each pixel which is why we model it as a binary classification task. For the results, we use pixel accuracy to evaluate the effect of the model. That is the proportion of pixels with correct classification in all pixels. It can be described by the following formula:

(4) $$\begin{array}{c} \text{piexl accuracy}=\frac{\sum \delta \left(y,\hat{y}\right)}{\text{image size}}. \end{array}$$

In the basic model and subsequent improved models, we use the above data sets division criteria and evaluation methods.

In the multiround training of the U-Net network, the model performance changes in Loss and Accuracy on the lung segmentation task, as shown in Figure 3.

It can be seen that the U-Net neural network performs relatively well on the two indicators of Loss and Accuracy. After about 20 epochs of training, the relevant indicators of the model have been iterated to a relatively good result. After 50 rounds of training, the accuracy of the model also reached more than 0.9. Although from the measurement of related indicators the model has achieved a good effect, in the actual imaging and segmentation process, we found that the generalization effect of the model is poor and the segmentation effect for other photos is not very good. We used the trained U-Net model to predict some of the X-rays of the test set and some of them were inferior. Here are some examples as shown in the X-ray film and its corresponding segmentation diagram in Figure 4.

Through the comparison between the actual original image and the predicted image, we can clearly see that the generalization effect of the model is not very satisfactory. For a part of the X-ray photos, after the lungs are completely segmented, some parts are also added background noise information, and for some pictures with poor original quality, the segmentation results are not satisfactory. Combined with the relevant analysis, we got the following explanation: in the photos presented by X-rays, we can intuitively see that there are obvious differences between the color of the lungs and the surroundings and the model has a better learning effect on this color difference but the learning is poor for features in other dimensions such as position and shape. Therefore, some background noises with similar color differences are not well distinguished.

The downstream DenseNet network adopts dense connections resulting in a large number of feature maps. In the case of multiple Dense Blocks and a large growth rate, it occupies a large amount of memory and is limited by relevant experimental conditions. With reducing the number of blocks while reducing the growth rate compared with the 121-layer DenseNet used in the original text, it uses a 4-layer block structure while the growth rate uses 24. The number of the block of the DenseNet-BC network we used in the experiment is 3, and the growth rate is 16. Therefore, the performance effect of the reduced DenseNet-BC in the downstream recognition task is also unsatisfactory; the related training situation is shown in Figure 5.

Although the two indicators of Loss and Accuracy are optimized in the trend from a global perspective, the optimization effect of the two is not obvious. The increase of Loss and Accuracy is within 10%, the increase in revenue is small, and there is still a big increase in the room for improvement. Judging from the final result, its level is far below that of professional radiologists.

From the perspective of related model indicators, the basic model has achieved good results on segmentation tasks but there is still a lot of room for improvement in the effect on classification tasks. We used the trained network to test some data and found the following problems:

1. Poor data quality: Because we use the public data set, the quality of the data is not very high. In the original image data, we obtained under the naked eye that the lungs of some pictures have low discrimination. The model based on this content learned is limited not enough to support the follow-up reasoning (Figure 6). Just like the two segmentation examples shown in the above figure, the left lung is not well segmented. After model training, the result still has such problems. By comparing the corresponding original images, we believe that such problems are caused by the data itself in X-ray imaging lung tissue and other tissues are not well distinguished by the naked eye; the data quality is not good; the knowledge that the model can learn from is limited and it cannot distinguish effectively.
2. Data imbalance: From the overall statistics, there is a great imbalance in the data set. Among the total image data of about 100000, the data related to pulmonary fibrosis only occupies a few thousand. Such an unbalanced data set is not friendly to the training model, the knowledge learned by the model is biased, the entire data distribution cannot be objectively evaluated, and the generalization ability is insufficient.
3. Insufficient model generalization ability: For a part of the test set data with better quality, we used the trained U-Net network to test and found that as shown in the figure below part of the lung, segmentation results are segmenting complete lungs, part of the background noise data is mixed with part of the background noise data, part of the task-irrelevant background is retained, and the actual effect of segmentation is not good. Based on other photos, we believe that the current model has learned the characteristics of the color dimension between adjacent areas. However, the model is not very effective for learning other dimensional features. For example, we believe that the model should also pay attention to the feature of the location. Normally in X-ray imaging, the lung tissue will be located in the middle of the photo rather than the edge. Therefore, when segmenting, the relevant images of the edge should be ignored (Figure 7).
4. Model representation ability is limited: We use the network structure of DenseNet-BC to complete downstream classification tasks but the limitation of computing power leads to the simplification of the network structure, reduces the number of blocks, reduces the growth rate, and leads to the model expressive ability not reached a very good level; the effect of classification has not reached the expectation, and there is still more room for optimization.

### 2.3. Predictive Model Using Divide and Conquer Strategy

In response to the problems of the basic model, we designed our own pulmonary fibrosis prediction model using a divide and conquer strategy. In upstream and downstream tasks, our proposed model has greatly improved over the basic model. At the same time, we have also optimized some problems in the prediction process of some basic models. According to the characteristics of the upstream and downstream tasks, we split it up and adopted the Attention-U-Net plus Inception-ResNet pulmonary fibrosis prediction model. Among them, the Attention-U-Net network is mainly used in upstream segmentation tasks. By adding the Attention structure on the basis of the U-Net network, we have achieved a greater improvement in the effect with a small increase in the amount of calculation. Inception-ResNet is used in downstream classification tasks. The two networks learn unbiased knowledge background through independent upstream and downstream training and they are used in the final lung fibrosis prediction task together.

#### 2.3.1. Attention: U-Net

The basic scheme performs well in the upstream lung segmentation part, and its index performance is better but the actual effect is still insufficient. We add the Attention structure to the basic U-Net network to improve and enhance the actual performance of the U-Net network. The U-Net network in the basic model retains part of the background noise in the actual segmentation process. In order to reduce the model's attention to background noise, we introduced an attention mechanism (Attention) and adopted the Attention-U-Net network structure for segmentation. The Attention mechanism [9–11] is based on the inspiration obtained from the human attention mechanism. When the human eye perceives the outside world such as watching photos movies and TV dramas, it tends to focus its attention on a certain part or a certain place to extract relevant information. Just like the camera focusing, you can use autofocus to blur the background or the portrait. The essence of these mechanisms is the distribution of attention coefficients. For task-related parts, a larger weight is assigned and the characteristics of this part are retained. For the parts that are irrelevant to other tasks, a small weight value is assigned to suppress. Therefore, it has a certain effect on improving the current model's attention to background noise.

Attention-U-Net was first proposed in 2018 [12] by introducing the corresponding Attention Gate structure on the basis of the U-Net model to retain task-related areas and suppress the task-independent areas so as to achieve better segmentation results Attention-U-Net's final network structure is shown in Figure 8.

Compared with the U-Net network structure, Attention-U-Net combines feature maps of different dimensions through the skip-connection structure after adding the gate signal of the Attention Gate to filter processing and adjusts the feature map of the Encoder to achieve effective information transmission and invalid information filtering. The principle can be understood as follows: after multiple downsampling, the model obtains the high-context information of the feature map, and this information gain can be used to filter the feature map under low-context conditions. Through the gate signal, the model can extract the core content of the information flow and eliminate redundant information. The related Attention Gate structure is shown in Figure 9.

The calculation formula of the weight matrix is as follows:

(5) $$\begin{array}{c} q_{att}^{l}=\phi^{T}\left(\sigma_{1}\left(W_{x}^{T}X_{i}^{l}+W_{g}^{T}g_{i}+b_{g}\right)\right)+b_{\phi },\\ \alpha_{i}^{l}=\sigma_{2}\left(q_{att}^{l}\left(x_{i}^{l},g_{i};\Theta_{att}\right)\right). \end{array}$$

At first, the feature map of the downsampling layer gets *W*_*g*_^*T*^*g*_*i*_ by convolution of 1 × 1 × 1, and the feature map of upsampling layer gets *W*_*x*_^*T*^*X*_*i*_^*l*^ by convolution of 1 × 1 × 1. After the results of the above two parts are added, the function is activated by Relu and then *ϕ*^*T*^(*σ*_1_(*W*_*x*_^*T*^*X*_*i*_^*l*^+*W*_*g*_^*T*^*g*_*i*_+*b*_*g*_))+*b*_*ϕ*_ is obtained by convolution of 1 × 1 × 1. Finally, the final attention weight matrix is obtained by activation of the Sigmoid function.

The attention weight matrix is used to adjust the information of the feature map. We multiply the attention matrix with the obtained feature map, readjust the images at different positions, and splice the adjusted images with the upsampling results as the input of the subsequent process.

#### 2.3.2. Inception-ResNet

In the basic scheme, we use the DenseNet-BC network to complete the downstream classification task but the final effect is not significant. The core idea of the DenseNet-BC network is to make the input of the current layer come not only from the output of the previous layer but also from all the previous layers by introducing a tight connection. This structure alleviates the problem of gradient disappearance and supports the further expansion of the network in depth. DenseNet and ResNet work in a similar way. Therefore, when the DenseNet network is not effective, we try to use the ResNet network for classification. ResNet (Residual Network) was put forward in 2015. Compared with DenseNet's dense connection, ResNet reduces the influence of gradient disappearance on neural network knowledge reasoning by introducing a layer-skipping connection between input and output, thus improving the expression ability of the model. Compared with DenseNet, residual connection in ResNet network can also improve network degradation which is similar to DenseNet. The contrast between residual connection and ordinary network connection is that for a hidden layer *H* in the network its input is *X* and its output is *H*(*X*), and ordinary neural networks can get the expression of function *H* through learning that is learning:

(6) $$\begin{array}{c} X⟶H\left(X\right). \end{array}$$

The residual connection focuses on learning the relationship between input and output; the following figure is a schematic diagram of the difference between the residual connection and the input and output of the common neural network. The residual unit accumulates the input and output of the unit by jumping layer connection (Figure 10).

Through the connection mode of jumping layers, the model learns the following relationship:

(7) $$\begin{array}{c} X⟶H\left(X\right)+X. \end{array}$$

ResNet-related series of networks are effective; the essence is the network depth which is further expanded by adding jump layer connection, and the expansion of the network depth improves the expression ability of the model. In addition to increasing the depth of the network, increasing the width of the network has a good optimization effect on the model-related indicators. This idea is adopted by Inception series networks [13] which increases the width of the model by adopting multiple parallel convolution operations at the same layer. In addition, multiple convolution kernels with different sizes can obtain image information with different scales, and the model synthesizes information with different scales, thus obtaining better prediction results. The structure of the Inception module is shown in Figure 11. By using multiple convolution kernels of different sizes in the same layer, the network can learn sparse and dense features which increases the adaptability of the network to scale. On the basis of the v1 version, Inception v2 converts the convolution kernel of 5 × 5 into two convolution kernels of 3 × 3 which reduces the parameter quantity and increases the depth of the network under the condition that the output feature map is unchanged and introduces the operation of Batch Normalization [14, 15] to prevent the model from overfitting. Its structure is shown in Figure 11.

By properly decomposing convolution and regularization, Inception v3 makes efficient use of huge parameters and it uses convolution and pooling in parallel to achieve dimension reduction and prevent the loss of relevant information. In Inception v4, the first few layers of feature extraction operations of the model are replaced by a Stem structure. The combination of the initiation network structure and ResNet network structure produces the initiation-ResNet series network, and we use the Inception-ResNet v2 structure as shown in Figure 12.

In the structure of the Inception-ResNet layer, the multiscale information of the image is extracted and fused by means of parallel convolution and layer-skipping connection while in the related layer of reduction the data is dimensionalized by means of parallel convolution and pooling operations which complement each other and avoid the loss of key information.

In the data preprocessing part of the network training, we also made partial optimization and we manually eliminated some data with poor quality. In addition, we also use data enhancement to improve the robustness of the model adding white noise to the input data randomly flipping left and right translating cropping, and so on. To solve the problem of unbalanced data sets, we increase the number of positive samples and reduce the impact of unbalanced data sets by upsampling. In the design of the loss function, we add different weights to balance the attention of the model to different types of data.

### 2.4. Results and Analysis

After improvement and optimization, the indexes of upstream and downstream tasks have been greatly improved. In the upstream segmentation task, the performance of the U-Net network is improved by adding the Attention structure, and the convergence speed of the Attention-U-Net network is faster when the final model accuracy is similar. From the actual renderings, the effect is better which better solves the problem that U-Net paid attention to background noise before. On the two indexes of Loss and Accuracy, the comparison between the Attention-U-Net network and the previous U-Net network is shown in Figure 13.

Through the measurement of Loss and Accuracy, we find that there is little difference in accuracy and result between them, but in convergence speed, Attention-U-Net is obviously better than the U-Net network. In addition, in the segmentation of actual pictures, we found that the effect of the Attention-U-Net model is better than that of U-Net, and the related actual renderings reveal such problems. We use the U-Net network and Attention-U-Net network to segment the same X-ray and the results are shown in Figure 14.

In the figure, the left side is the segmentation map of lung tissue by the U-Net network while the right side is the segmentation map using Attention-U-Net. It can be seen intuitively that the actual segmentation effect of the Attention-U-Net network is better.

For downstream tasks after using ResNet instead of DenseNet, the effect of the two pairs is as shown in Figure 15.

It can be seen that after using the ResNet network structure the Loss and Accuracy indicators have been significantly improved. We used the ResNet-34 network to predict pulmonary fibrosis. Besides, we added L2 regular term for improving the problem of excessive fluctuations in the loss function. In addition, on the basis of ResNet-34, we further increase the number of layers of the network that is using ResNet-34+L2 regular term coefficients and ResNet-50+L2 regular term coefficients to predict lung fibrosis each; the comparison effect of the model on this task is shown in Figure 16.

It can be seen from the figure that the ResNet series models perform better than the DenseNet network in downstream classification tasks. Moreover, the performance of the ResNet network has been improved with the increase in depth and the speed of convergence has further increased. The ResNet-50 model used finally has reached a good level from the index point of view.

The Inception-ResNet v2 network which integrates multiscale information and layer-jumping connections that have grown in the width and depth of the model has achieved better results in downstream prediction tasks. We use the Inception-ResNet-v2 network to perform related training on the segmented X-ray data set, and the related training index changes are shown in Figure 17.

As can be seen from Loss and Accuracy, the convergence of the Inception-ResNet v2 model appears to be more gradual, and the final result is even better. We compared the ResNet DenseNet and other networks we have used in Inception-ResNet v2 horizontally. The effect comparison chart is shown in Figure 18.

It can be clearly seen from the figure that the Inception-ResNet v2 network surpasses the previous ResNet-related methods in terms of convergence speed and accuracy and has better results. Our optimization has also achieved better results, and the accuracy of each method is about 0.9 which has a certain generalization and application value.

Through the horizontal and vertical comparison, the combination of the Attention-U-Net model and the Inception-ResNet v2 model we proposed achieves the best results in the prediction of lung fibrosis based on X-rays.

## 3. Conclusion

As a tumor-like disease, pulmonary fibrosis disease has no effective treatment methods and drugs. The main purpose of existing drugs is to prolong the life of patients. The length of life depends largely on the time for diagnosis and treatment. Early diagnosis and early treatment will better guard life.

As a common clinical imaging data, X-ray has a very good auxiliary role in the auxiliary diagnosis of various diseases. Through related images, the tissues and organs in the body can be visually observed to quickly locate the lesion and confirm the case.

Based on the X-ray film, we proposed the upstream Attention-U-Net segmentation and downstream Inception-ResNet v2 solution models which achieved relatively good results in experiments, and the relevant diagnostic level is close to that of professional imaging doctors. Because we added some new data on the basis of the data set chest X-ray 14, we use ResNet-50 [3] and DenseNet-121 [4], respectively, to compare with the Inception-ResNet-v2 method. We use the accuracy in the test set for comparison. Using 20% of the data set as the test set, we found that the classification accuracy of ResNet-50 was about 89% while the accuracy of Inception-ResNet v2 was 93% which was greatly improved compared with ResNet. Because DenseNet occupied too many resources, we cut the network appropriately and the results are not included in the scope of comparison.

Figure 18 shows the continuous change of relevant loss of the model during training. It can be found that the Inception-ResNet v2 model is also superior to other methods in terms of convergence effect. At present, the transformer has shown amazing results in image classification segmentation and other tasks. In the follow-up work, we will try to use relevant technologies to improve the performance of pulmonary fibrosis prediction tasks.

Due to the upsampling and downsampling of our data set, the imbalance of distribution is adjusted. Therefore, even if the model reaches a level higher than that of human doctors, it still cannot be directly applied to the actual scene. We try to work with radiologists to improve the accuracy and speed of the model in the real scene.

In summary, this article starts from the background of pulmonary fibrosis prediction and completes the whole process from data processing model design to final deployment. For pulmonary fibrosis, a predictive solution model based on a deep neural network is proposed. However, due to the limited amount of computing, power and data obtained the complexity of the model and the final effect still have room for optimization. Later, it can be improved by deploying larger models to apply to related data sets. In addition, in view of the insufficiency of medical imaging-related data, we can strengthen cooperation with professional radiologists, expand and improve our own data sets or design-related marking procedures, and use NLP-related technology to learn from professional doctors' diagnosis and treatment process; the corresponding data is marked and saved which supports the realization of a more comprehensive and accurate prediction model of pulmonary fibrosis.

## Figures and Tables

**Figure 1:** Dense connection diagram.

**Figure 2:** DenseNet BC network structure diagram.

**Figure 3:** U-net network index change chart.

**Figure 4:** Comparison of segmentation effect.

**Figure 5:** Change chart of DenseNet BC network-related indicators.

**Figure 6:** Comparison of original image and segmentation image.

**Figure 7:** Segmentation effect diagram.

**Figure 8:** Attention—U-Net network structure diagram.

**Figure 9:** Attention Gate structure diagram.

**Figure 10:** Diagram of the difference between residual connection and ordinary connection.

**Figure 11:** Inception module.

**Figure 12:** Inception-ResNet v2 network diagram.

**Figure 13:** Attention-U-Net and U-Net effect comparison chart.

**Figure 14:** Comparison chart of lung segmentation effect.

**Figure 15:** Comparison of DenseNet-BC and ResNet34.

**Figure 16:** ResNet-related model and DenseNet effect comparison chart.

**Figure 17:** Inception-ResNet v2 network-related indicators.

**Figure 18:** Comparison of various models in X-ray classification tasks.

## Data Availability

In the actual application, in addition to the public data set, this paper uses some real data from the hospital. This part of the data is currently under embargo while the research findings are commercialized.
